The article "“Worse than I anticipated” or “This isn’t so bad”?: The impact of affective forecasting accuracy on self-reported task performance" was published in 2020. Journal: PLoS One.

# “Worse than I anticipated” or “This isn’t so bad”?: The impact of affective forecasting accuracy on self-reported task performance

**DOI:** 10.1371/journal.pone.0235973

**Published:** 2020-07-13

**Authors:** Seth Kaplan, Carolyn Winslow, Lydia Craig, Xue Lei, Carol Wong, Jill Bradley-Geist, Martin Biskup, Gregory Ruark

**Affiliations:** 1 George Mason University, Fairfax, Virginia, United States of America; 2 University of California, Berkeley, California, United States of America; 3 University of Colorado, Colorado Springs, Colorado, United States of America; 4 U.S. Army Research Institute for the Behavioral and Social Sciences, Fairfax, Virginia, United States of America; University of Lleida, SPAIN

## Abstract

Various motivational theories emphasize that desired emotional outcomes guide behavioral choices. Although motivational theory and research has emphasized that behavior is affected by desired emotional outcomes, little research has focused on the impact of anticipated feelings about *engaging in behavior*. The current research seeks to partly fill that void. Specifically, we borrow from affective forecasting research in suggesting that forecasts about engaging in performance-relevant behaviors can be more or less accurate. Furthermore, we suggest that the degree of accuracy has implications for self-reported task performance. To examine these ideas, we conducted two studies in which individuals made affective predictions about engaging in tasks and then later reported how they actually felt during task engagement. We also assessed their self-reported task performance. In Study 1, 214 workers provided affective forecasts about upcoming work tasks, and in Study 2, 185 students made forecasts about studying for an exam. Results based on polynomial regression were largely consistent across the studies. The accuracy of the forecasts did not conform to the pattern of affective forecasting accuracy typically found outside the performance domain. Furthermore, anticipated and experienced affect jointly predicted self-reported task performance in a consistent manner. Collectively, these findings suggest that taking into account anticipated affect, and its relationship with later experienced affect, provides a more comprehensive account of affect’s role in task performance.

## Introduction

A fundamental tenet in various theories of human motivation and well-being is that, all else being equal, people prefer positively-valenced emotional states to negative ones [1]. As such, choices often reflect a desire to bring about these positive states [2]. What recent research has made evident, though, is that the outcomes of these choices often do not yield the emotions we hoped or feared they would. Research on “affective forecasting” documents systematic inconsistencies about future anticipated affective states. These inaccuracies manifest for both positive and negative anticipated affect. They also result across a range of life outcomes, ranging from commonplace (e.g., making illogical investment decisions due to overestimating potential emotional reactions [3]) to life-changing ones (e.g., receiving an HIV diagnosis [4]). In addition to their theoretical value, these findings have practical significance with respect to how people make life choices [5, 6, 7].

Largely lost from this discussion, though, is the recognition that one not only anticipates emotion about upcoming choices and outcomes but also about *engaging in effortful behaviors*. To illustrate this point, we offer the example of an employee writing a report. Task motivation—and subsequent performance—certainly may be a function of the value of the outcomes that would follow from a complete and well-written report (e.g., praise from one’s supervisor, increased self-worth, etc. [8]). However, motivation and resultant performance is also likely influenced by the employees’ expectations about how they will feel while actually doing the writing (not only feelings resulting from the outcomes of having done so).

In the current research, we examine the implications that such (in)accuracy may have for performance on the focal task. Thus, for example, what is the impact on task performance when engaging in this seemingly aversive behavior/activity is not as onerous as anticipated, or is perhaps even pleasant? Alternatively, what happens when engaging in the behavior is even more aversive than we had forecasted it to be? Just as we now know that intuition about the impact of outcome of life choices and various life circumstances often are in error [9], so too may be predictions about engaging in task work.

In the following pages, we elaborate on whether and in which form (in)accuracy in these forecasts may benefit (versus hurt) self-reported performance on the relevant task. After this Introduction, we present two studies testing the propositions we develop below.

### Affective forecasting and behavioral outcomes

Affective forecasts represent predictions about future emotional states. Research on affective forecasting primarily focuses on the factors that contribute to the accuracy of predictions about future emotional states (for reviews, see [9, 10]). Within this literature, many studies explore affective forecasts when people consider and experience discrete (and sometimes uncontrollable) events or life outcomes (such as being denied tenure or receiving a diagnosis of a disease). Other studies examine forecasting (accuracy) when people make choices and decisions. These scenarios include choices about which social relationships to engage in [11], health-related matters [12], and consumer-related choices [2]. As is clear from these examples, the “behaviors” of interest in this literature mostly have been decisions about particular outcomes or discrete decisions, not behaviors requiring sustained effort to accomplish a task.

As with much of the affect literature, research on affective forecasts incorporates the notion that feeling states have evolved to motivate behavior [13]. Where affective forecasting research differs from other relevant accounts is in regard to just how affect functions. Specifically, affective forecasting prioritizes *anticipated affect*, versus *experienced affec*t, in guiding the instantiation of behavior.

Consistent with a proposed motivational significance of *anticipated* affect, Baumeister et al. [14] have suggested that the traditional view of the affect-behavior relationship is misguided or, at a minimum, incomplete. According to their emotion-as-feedback theory, *anticipated* emotion (not resultant or “in-the-moment” emotion) is the proximal cause of behavior. Studies indeed show that anticipatory feelings about how one will feel after making certain choices or performing certain discrete behaviors (e.g., helping someone) better predict the choice/behavior than do in-the-moment feelings [15].

### Affective forecasting about engaging in task behavior

As summarized above, the affective forecasting literature primarily focuses on anticipated feelings about discrete *outcomes* that are beyond one’s control or about outcomes resulting from particular choices or behaviors. Largely neglected in this corpus of work is the recognition that we spend much of our time performing effortful and prolonged goal-directed behaviors. Unlike the scenarios that have been the focus of the affective forecasting literature, these behaviors generally have no obvious outcome other than their completion. Representative behaviors include many work tasks (e.g., writing emails, interacting with clients), housework (e.g., cleaning, ironing), and caring for and helping other household members (e.g., helping children with homework) [16]. This oversight in the literature is perhaps surprising given two research conclusions, namely, 1) that effortful behavior often is an emotional experience [17], and 2) that planning and strategizing are the most commonly reported functions of future-oriented thoughts [18]. Given these conclusions, studying the implications of affective forecasts about task behavior seems worthwhile.

### Development of research propositions

We develop the study propositions below. We draw on affect-as-information theory [19, 20, 21] to support and guide the following discussion. According to affect-as-information theory, people use their affect as information in making evaluative judgments. At the most basic level, positive affect (PA) signals a safe environment and negative affect (NA) signals a threatening one [21]. Especially relevant to the current theorizing, affect can serve as information about *progress* or *success* regarding task behavior [19]. That is, affect can impact interpretations of how well one is doing in terms of moving toward task goals [22]. Seen in this light, affect represents a motivational input that is subsequently interpreted.

We extend this research by examining the motivational influence of the interplay between anticipated and experienced affect. As affect varies in intensity and valence [23, 24] different types of affective discrepancies are possible. Discrepancies can exist/vary in terms of magnitude (i.e., the size of discrepancies between anticipated and experienced affect) and/or valence (here, when experienced PA or NA, respectively, is higher or lower than anticipated). In turn, different types of discrepancies may result in different performance effects. As elaborated upon below, the present study focuses on identifying the types of affect discrepancies that are associated with *enhanced* self-reported performance

#### The interplay between anticipated and experienced affect

We present three plausible possibilities regarding the interplay between anticipated and experienced affect and task performance:

*Proposition 1*: *Congruence* between anticipated and experienced affect will be associated with enhanced self-reported task performance;

*Proposition 2*: *Positive incongruence* between anticipated and experienced affect (i.e., Feeling “better” than anticipated) will be associated with enhanced self-reported task performance;

*Proposition 3*: *Negative incongruenc*e between anticipated and experienced affect (i.e., Feeling “worse” than anticipated) will be associated with enhanced self-reported task performance.

We first consider the possibility that *congruenc*e between anticipated and experienced affect helps self-reported performance (Proposition 1). In this study, we use Watson’s [24] dimensions of PA and NA. Thus, congruence here means that the level of anticipated PA or NA is equal to (or approximately equal to) the level of experienced PA or NA (Experienced PA = /≈anticipated PA and Experienced NA = /≈ anticipated NA).

Our reasoning begins with the fact that attentional resources needed for effective task performance are limited [25]. Attending to, and possibly regulating, discrepant emotional experiences would draw from that attentional reservoir, thereby potentially degrading performance [26]. When experienced affect is consistent with anticipated affect, there is no discrepancy to hijack additional mental resources, thereby leaving more attentional focus to the present task.

Unlike positive and negative incongruence (discussed next), the congruence proposition states that any deviation is detrimental, irrespective of the direction of the deviation or the valence of the affect (i.e., PA or NA). Thus, anticipating that a task will be quite distasteful and then finding it less distasteful than anticipated, for instance, also should draw attentional resources and hinder performance.

The other two possibilities suggest that discrepancies between anticipated and experienced affect will benefit self-reported performance. The basic idea that discrepancies may be functional derives from the widespread documentation of systematic inaccuracies in affective forecasting [9]. Miloyan and Suddendorf [27] suggest that a primary role of affective forecasting errors is behavior regulation. As those authors note, discussions of affective forecasting errors largely have focused on the costs of such inaccuracy. However, if one accepts that affect has evolved to serve motivational purposes, discrepancies in forecasts also should be beneficial.

One type of discrepancy is what we label *positive incongruence*, or when people generally feel “better” than anticipated. Defined specifically, positive incongruence is when anticipated NA exceeds experienced NA (anticipated NA > Experienced NA), or when experienced PA exceeds anticipated PA (Experienced PA > anticipated PA). As noted above, affect can serve as information about progress or success during task behavior; here we suggest that affect discrepancies can serve similar purposes. Specifically, positive incongruence may enhance performance by signaling progress and competence, and, in turn, facilitate continued motivation and task effort [28]. Similarly, feeling more positively than anticipated may promote performance through persistence, as individuals generally strive to engage in and maintain pleasant affective states and avoid unpleasant ones [2]. Of note, this PA also could result from affect incidental to the task itself (e.g., the social context or what happened previously that day).

The final possibility we consider is *negative incongruence or* when people generally feel “worse” than anticipated. Defined specifically, *negative incongruence* is when experienced NA exceeds anticipated NA (Experienced NA > anticipated NA), or when anticipated PA exceeds experienced PA (anticipated PA > Experienced PA). Negative incongruence may facilitate performance by signaling *lack* of progress and/or *in*competence. In turn, such perceptions may facilitate continued motivation and increased effort. Thus, consistent with affect-as-information theory, it is plausible that either positive or negative incongruence could result in enhanced performance.

*Research Question*: Under which affective forecasting scenario will self-reported task performance be enhanced: *congruence*, *positive incongruence*, or *negative incongruence*?

### Overview of studies

To address this research question, we conducted two studies examining real-world task performance. We employ the same paradigm in both studies. Individuals first report their anticipated affect about engaging in the focal task/activity and subsequently report their experienced affect. This allowed for examining the joint role of anticipated and experienced affect on self-reported performance. We describe the Study 1 Method below.

## Study 1 method

### Data and sample

This research was approved by the Institutional Review Boards of George Mason University and University of Colorado Colorado Springs. It was also approved by the US Army Research Institute Human Research Protection Official Review. Participants in the eastern U.S. were recruited through Craigslist and received compensation in the form of Amazon gift cards. Participants were informed that there was no foreseeable risk associated with their participation and they were free to withdraw at any time. All participants provided informed consent before participating. A total of 264 people responded to the Time 1 survey and at least one follow-up survey (i.e., about later experienced affect). The final sample consisted of 767 usable tasks/activities provided by 214 participants, who represented a wide variety of industries, including health care, education, food services, information technology, and manufacturing. The average age of participants was 30.52 (*SD* = 8.77), and 52.88% were female. The average job tenure and organizational tenure were 3.43 years (*SD* = 3.66) and 4.55 years (*SD* = 5.05), respectively. Racial and ethnic composition of the sample was 77.10% White, 10.28% Black/African American, and 10.28% Asian, with the remainder representing other groups.

Online surveys were administered across multiple time points. At time 1, participants listed and made ratings about five work tasks/activities anticipated to occur during the upcoming workweek. Participants were required to choose work events occurring at least two days after the day they completed the baseline survey (to eliminate any possible recall effects). During the following workweek, participants completed “post-activity” surveys on each day when an at least one of the activities about which they had made forecasts was anticipated to occur. Participants were able to complete post-activity surveys until midnight of the day in which the task/activity was to occur. A few participants misunderstood instructions on the baseline survey and listed events occurring beyond that workweek–with a maximum of 12 days occurring between the baseline survey and the final post-survey. Because conclusions did not change without these data points, we retained them.

### Measures

#### Time 1 measures

Participants were asked to think of five different work-related activities they were likely to experience during the next work week. Because we hoped to sample various types of activities, participants were told these could be either typical, regularly occurring work activities or more unusual, infrequently occurring activities. Participants listed these activities and provided brief descriptions of each activity. For descriptive purposes, we also asked participants to report the frequency with which they engage in each of the activities at work using a 5-point scale from “Very rarely (once a month or less)” to “Very often (most days or multiple times per day)”. This was meant to capture familiarity.

#### Affective forecasts

Participants reported their anticipated affect for three NA states (anger/annoyance, anxiety/worry, and tiredness/fatigue) and two PA states (happiness/pleasure and relaxation/comfort) during each upcoming activity. Specifically, after listing each activity (and providing the day and time of its upcoming occurrence), participants were asked to rate, “the extent to which you anticipate experiencing each of the following emotions the next time you engage in this event/activity.” We chose these five states based on Mignonac and Herrbach’s [29] study of common workplace affective experiences. Responses were made on a 5-point Likert scale ranging from 1 (“Not at all”) to 5 (“A great deal”). We analyzed each emotion state separately and also created scale scores for NA and PA. Coefficient alpha reliability = .75 for the NA scale and .88 for the PA scale.

#### Experienced affect

In post-activity surveys, participants first reported whether they engaged in the anticipated/scheduled activity. Participants also indicated the actual time and total duration of each activity. We eliminated activities that did not occur as scheduled (< 5% of activities). Next, the same items as above were used to measure experienced affect during the activity that had just occurred, “I was feeling…” (α = .78 for NA, α = .85 for PA). Self-reported performance was measured using the item “How well do you think you performed during this particular event/activity?” using a 1 (“Very poorly”) to 4 (“Very well”) scale.

### Study 1 results

#### Descriptive results regarding affective forecasting accuracy

Fig 1 presents the means, standard deviations, and correlations for the study variables. Given that this is the first study of which we are aware examining the accuracy of task-related affective forecasts, we first present descriptive results regarding the accuracy of the forecasts. To assess accuracy, we first calculated discrepancy scores between anticipated and experienced affect (i.e., anticipated—experienced affect or “directional” accuracy, a measure of *incongruence* as noted above). The directional discrepancies approximated normal distributions, with around half of the scores distributed near the central point (proportions of discrepancies within -0.5 to 0.5 were: PA: 62%, NA: 71%, happiness: 45%, relaxation: 46%, anger: 51%, anxiety: 52%, and tiredness: 45%), with the remaining discrepancy scores symmetrically distributed on the two sides. The frequency distributions are available upon request from the corresponding author. This trend was consistent for the five discrete emotion states as well as for PA and NA. Thus, there was not a tendency to systematically forecast work tasks as being more or less aversive or pleasant than anticipated (positive and negative incongruence). Follow-up regression analyses for each of the discrete emotions (using robust standard errors to account for the nested data structure; i.e., episodes within persons) confirmed that there was not an obvious trend to overpredict or underpredict these emotions.

**Fig 1:** Study 1 descriptive statistic and correlations. N = 767. Correlations are at the event level. All correlations are significant at p < .01. Alpha coefficients are displayed on the diagonal in parentheses.

We also examined the absolute accuracy (i.e., not taking into account the direction of discrepancies). To do so, we calculated the absolute values of the discrepancy scores involving anticipated versus experienced affect for all the five discrete emotions and PA and NA. The descriptive statistics showed that the absolute discrepancies for both PA (mean = .68, SD = .70) and NA (mean = .53, SD = .55) were relatively small. Following suggested practice [30], we standardized anticipated and experienced affect. Shanock et al. [30] suggested the use of .5 SD as a criterion to determine accuracy. Overall, about half of the absolute discrepancy scores were less than .5 SD units (happiness: 45%, relaxation: 45.9%, anger: 51%, anxiety: 52.2%, and tiredness: 44.9%). These results suggested a fair degree of accuracy but also variability in accuracy.

#### Results for primary research question

Before testing the primary research question, two authors independently coded the data to ensure that each activity was relevant to task (i.e., job) performance. Initial agreement between the coders was 98% and any discrepancies were resolved through discussion. The coding revealed that 17 of the 767 reported activities (2.22%) were performance irrelevant and thus were excluded from the following analyses. Examples of performance irrelevant activities included “Walk to the coffee shop,” “Eating lunch with coworkers,” and “Office party.”

To address the primary research question, we used polynomial regression with response surface analysis [31]. The nested structure of the data (episodes within persons) required the use of Hierarchical Linear Modeling (HLM) for the polynomial regressions. In these models, we estimated random effects for the intercept (b_0_) and each of the linear effects (b_1_ and b_2_). To aide with interpretation and to reduce multicollinearity, prior to the analysis, we scale-centered the predictors by subtracting the scale midpoint (i.e., 3 on a 5-point scale).

The main emphasis in polynomial regression is on the response surfaces and their values. We examined the slope and curvature of two specific lines in the response surfaces [30]. The “line of perfect agreement” captures the relationship between the predictors (anticipated affect and experienced affect) and the outcome variable (self-reported performance) when the predictors are exactly equivalent (X = Y). The “line of incongruence” captures the same relationship when the predictors are exactly opposite (X = -Y).

Because the conclusions for the main research question were identical for the three respective negative emotions and for the two positive ones, respectively, we focus on the NA and PA scale scores below. Turning first to the response surface results for PA (Fig 2), the line of agreement indicates that self-reported performance is higher when both anticipated and experienced PA are high versus when both predictors are low (*a*_1_ = .28, *SE* = .03, *t* = 9.52, *p* < .001). Thus, self-reported performance benefits when employees forecast feeling positively about engaging in the upcoming task and feel positively when so engaged. This line is also non-linear (*a*_2_ = .04, *SE* = .02, *t* = 2.63, *p* = .009), meaning that the relationship is convex or upward curving. The latter finding means that self-reported performance increases at a higher rate as both anticipated and experienced PA become higher.

**Fig 2:** Response surface area wherein self-reported performance is predicted by the anticipated—experienced positive affect discrepancy (Study 1). Of note, when conducting polynomial regression, we scale-centered the predictors by subtracting the scale midpoint to reduce multicollinearity and aide interpretation. Each of the predictors evaluated in both studies were measured on a 5 point scale as noted in the Method sections; therefore we subtracted 3 from each predictor value, resulting in the values -2 to 2 in the along the X- and Y-axes in Figs 2–7. The variables on the Z- axes in Figs 2–7 are not centered and reflect the original 5-point Likert scale responses used (with the exception of time spent studying in study 2, which was assessed in minutes).

Next, regarding misfit, the line of incongruence indicates that self-reported performance is higher when experienced PA is higher than anticipated PA (i.e., underprediction), compared to when experienced PA is lower than anticipated PA (i.e., overprediction; *a*_3_ = -.10, *SE* = .04, *t* = -2.33, *p* = .020). Curvature along the line of incongruence was significant at a trend level (*a*_4_ = .06, *SE* = .04, *t* = 1.63, *p* = .103). Here, upward curvature along the line of incongruence suggests that self-reported performance increases more sharply as the degree of the discrepancy grows between anticipated and experienced PA. In sum, these results support both the congruence proposition and the positive incongruence notion for PA: affective experiences that are anticipated to be positive and are indeed positive tend to be associated with higher levels of self-reported performance. These ratings of performance benefit even further when PA exceeds expectations.

With regard to the response surface results for NA (Fig 3), the line of agreement indicates that self-reported performance is higher when both anticipated and experienced NA are low versus when both predictors are high (*a*_1_ = -.32, *SE* = .06, *t* = -5.80, *p* < .001). In contrast with the results for PA, the curvature of the line of agreement for NA was not significant (*a*_2_ = .01, *SE* = .03, *t* = .42, *p* = .673). Regarding misfit, the line of incongruence indicates that self-reported performance is higher when experienced NA is lower than anticipated NA (i.e., overprediction), compared to when experienced NA is higher than anticipated NA (i.e., underprediction; *a*_3_ = .23, *SE* = .08, *t* = 2.82, *p* = .005). Last, curvature along the line of incongruence also approached statistical significance (*a*_4_ = .10, *SE* = .06, *t* = 1.76, *p* = .078). Upward curvature along the line of incongruence suggests that self-reported performance increases more sharply as the degree of the discrepancy grows between anticipated and experienced NA. Collectively, these results also support the congruence and the positive congruence propositions. Ratings of performance are enhanced when NA is anticipated to be low and then is low; they are enhanced further when experienced NA is even lower than anticipated.

**Fig 3:** Response surface area wherein self-reported performance is predicted by the anticipated—experienced negative affect discrepancy (Study 1).

### Study 1 discussion and study 2 overview

Study 1 examined the accuracy and self-reported task performance implications of affective forecasts in a naturalistic field sample with multiple types of jobs. Descriptive results evaluating forecasting accuracy indicated that there was considerable variability in the accuracy of these forecasts, and that this variability was normally distributed. Also, in many cases, employees, *did* accurately predict how they would feel while performing work-related tasks. Notably, these results largely differ from the dominant findings in the affective forecasting literature.

With regard to the primary research question, findings provide initial support for both the *congruence* and *positive incongruence* propositions for both PA and NA. Specifically, for PA, self-reported performance is enhanced when PA is anticipated to be high and then is high and is further enhanced when PA is higher than anticipated. Likewise, for NA, self-reported performance is enhanced when NA is anticipated to be low and then is low and is enhanced further when experienced NA is even lower than anticipated.

Taken together, the first study represented an initial exploration of how task-related affective forecasts influence self-reported work performance. We sought to replicate and expand upon this initial study with a second study. Study 2 extends Study 1 in two key ways–by examining ratings of task performance within a different context and population, and by exploring more process-oriented indicators of performance.

Regarding study context/population, whereas Study 1 included a wide variety of occupations, tasks, and work environments, we intentionally narrow the context in Study 2 to a particular population (students) performing a particular task (studying/preparing for a course exam). This narrowing allowed us to examine the research questions in a more focused way by eliminating much of the variability in task type.

It also helped in disentangling affect about engaging in the task from affect about success on it. Specifically, because Study 1 asked about “performance”, affect ratings (both anticipated and experienced) may have reflected some combination of thoughts/reactions about *completing* the task and about *perceived success* performing it. In Study 2, we sought to isolate the processes associated with completing an intermediary task (studying for an exam) with participants lacking objective feedback about their success in performing the ultimate task (e.g., taking the exam for which they were studying). Accordingly, participants in Study 2 made predictions about goal-directed behaviors (while studying for an exam) rather than about overall task performance itself as was done in Study 1.

## Study 2 methods

### Data and sample

This research was approved by the Institutional Review Boards of George Mason University and University of Colorado Colorado Springs. It was also approved by the US Army Research Institute Human Research Protection Official Review. Undergraduate students from a large, public university located in the eastern U.S. participated in this study and received compensation in the form of course credit and/or a monetary reward. Participants were informed that there was no foreseeable risk associated with their participation and they were free to withdraw at any time. All participants provided informed consent before participating. A total of 185 complete responses (those who filled out all of the surveys as described next) were used in the analyses. The average age of participants was 21.20 (*SD* = 2.90), and 62.73% of participants were female. The racial and ethnic composition of the sample was 34.12% White, 37.83% Asian, and 8.64% Black/African American, with the remainder of the sample representing other groups.

Online surveys were administered across multiple time points. In the first survey, participants anticipated how they would feel while studying for an upcoming exam that was at least a week away. Participants made forecasts about specific study episodes they had planned that were within three days of the upcoming exam. Three (versus more) days were chosen given evidence that most studying for college exams occurs in the days immediately preceding the exams [32]. Because variables such as degree of familiarity with the exam format potentially could influence performance on the first exam for a given course, participants were asked to provide information for exams other than their first one in that course. In the second set of surveys, participants reported experienced affect and completed measures of goal-directed behaviors while studying for the exam.

### Measures

#### Affective forecasts

One week prior to the exam, participants made affective forecasts about how they would feel during specific planned study episodes for that exam. Affect was measured using the Positive and Negative Affect Schedule (PANAS) [33]. Participants were asked to indicate the extent to which they would feel each of the 20 PANAS emotions (10 each for PA and NA) while studying for the exam. Responses were made on a 5-point Likert-type scale ranging from 1 (“Not at all”) to 5 (“Extremely”). α for anticipated PA and for anticipated NA both = .89.

#### Experienced affect

Participants were sent e-mail reminders on the day of planned study episode to report their experienced affect. Specifically, participants indicated the extent to which they had experienced each emotion while studying. Experienced affect also was assessed using the PANAS [33]. Coefficient alpha reliability for experienced PA and NA were .90 and .91, respectively.

*Goal-directed behaviors*. Goal-directed behaviors are defined here as actions that involve self-regulation and facilitate completion of task-related goals. In this study, we examined attentional focus, problem-focused coping, and time spent studying.

Attentional focus refers to the narrowing of one’s focus to limited stimuli [26]. It was assessed using a four-item scale developed by Ghani and Deshpande [34] which was adapted to the context of studying. While studying, students indicated the extent to which they were engrossed and absorbed in the activity, using a 5-point Likert-type scale ranging from 1 (“Not at all”) to 5 (“Extremely”; α = .86.)

Problem-focused coping refers to efforts for reducing the negative consequences of stressors through an active focus on problem resolution [35]. It was assessed using seven items adapted from the problem-focused coping scales of the *Student Coping Instrument* (SCOPE) [36]. Items from three different subscales were used: Academic Planning (e.g., “I thought hard about what steps to take”), Active Study Coping (e.g., “I used a study guide”), and General Active Coping (e.g., “I took action to make progress”). Participants were asked to respond using a 5-point Likert scale ranging from 1 (“Strongly disagree”) to 5 (“Strongly agree”). Coefficient alpha reliability = .70.

Time spent studying was recorded as the total (cumulative) number of minutes students self-reported spending studying for the exam in the three days leading up to the exam. Including this outcome also speaks to the theoretical mechanisms at play. If feeling better than expected resulted in less time studying (consistent with the Study 1 findings), this result would imply that such a discrepancy is associated with more efficient behavior/processing, at least for a cognitively demanding task like studying.

### Study 2 results

Given that Study 2 was intended to serve as a replication study in a different context, we followed the same general analytical procedures, again evaluating the accuracy of affective forecasts, followed by examining the joint effects of anticipated and experienced PA and NA on self-reported performance (in this study, the goal-directed behaviors, which can be considered more proximal indicators of performance).

#### Descriptive results regarding affective forecasting accuracy

Table 1 presents the means, standard deviations, and correlations for all study variables. With regard to the accuracy of task-related affective forecasts, directional discrepancies again closely approximated normal distributions. The majority of scores were located near the central point (proportions of discrepancies within -0.5 to 0.5 were: PA: 66%, NA: 65%), with the remaining discrepancy scores approximately symmetrically distributed. The frequency distributions are available upon request from the corresponding author. These findings indicate that, as in study 1, there was not a tendency to systematically over- or underpredict PA or NA experienced while studying.

**Table 1:** Study 2 descriptive statistics and correlations.

	Mean	SD	1	2	3	4	5	6
1. Anticipated Positive Affect	2.66	.77	.*89*					
2. Anticipated Negative Affect	2.38	.82	.11	.*89*				
3. Experienced Positive Affect	2.71	.77	.72	.06	.*90*			
4. Experienced Negative Affect	2.32	.74	.21	.74	.21	.*91*		
5. Attentional Focus	3.15	.74	.38	-.01	.57	-.01	.*86*	
6. Problem-focused Coping	3.61	.57	.31	-.02	.53	.03	.47	.*70*
7. Time Spent Studying	595.75	524.76	.20	.16	.33	.25	.28	.29

N = 185. Correlations greater than |.16| are significant at *p* < .05; correlations greater than |.20| are significant at *p* < .01. With a Holm Bonferroni correction, correlations greater than |.20| are significant at *p* < .05. Alpha coefficients are displayed on the diagonal in italics. Time spent studying is in minutes.

Regarding absolute accuracy, descriptive statistics indicated that discrepancies between anticipated and experienced affect were relatively small for both PA (mean = .45, *SD* = .36) and NA (mean = .43, *SD* = .36). Furthermore, about 65% of the absolute discrepancies were less than .5 SD units, suggesting a fair amount of accuracy, but also some variability.

#### Results for primary research question

Next, as in Study 1, we used polynomial regression with response surface analysis [31] to examine the relationships between affective forecasting accuracy (i.e., anticipated affect and experienced affect) and goal-directed behaviors. The response surfaces for PA predicting focus, coping, and time spent studying is shown in Figs 4–6. The line of agreement indicates that focus, coping, and time spent studying are higher when both anticipated and experienced PA are high versus when both predictors are low (for focus, *a*_1_ = .51, *SE* = .15, *t* = 3.39, *p* = .001; for coping, *a*_1_ = .33, *SE* = .05, *t* = 6.50, *p* < .000, for time spent studying, *a*_1_ = 253.93, *SE* = 57.99, *t* = 4.38, *p* = .000). Thus, in support of the congruence proposition, goal-directed behaviors increase when employees forecast feeling positively about engaging in the upcoming task and feel positively when so engaged. Curvature along this line was significant for time spent studying (*a*_2_ = 157.59, *SE* = 54.92, *t* = 2.87, *p* = .005), but not significant for focus and coping (for focus, *a*_2_ = -.06, *SE* = .07, *t* = -.852, *p* = .395, for coping, *a*_2_ = -.06, *SE* = .04, t = -1.368, p = .173). These findings indicate that the relationship is convex or upward curving for time spent studying, meaning that time spent studying increases at a higher rate as both anticipated and experienced positive affect increase.

**Fig 4:** Response surface area wherein attentional focus is predicted by anticipated—experienced positive affect discrepancy (Study 2).

**Fig 5:** Response surface area wherein problem-focused coping is predicted by anticipated—experienced positive affect discrepancy (Study 2).

**Fig 6:** Response surface area wherein time spent studying is predicted by anticipated—experienced positive affect discrepancy (Study 2).

Next, the line of incongruence indicates that focus, coping, and time spent studying are higher when experienced PA is higher than anticipated PA (i.e., underprediction), compared to when experienced PA is lower than anticipated PA (i.e., overprediction; for focus, *a*_3_ = -.66, *SE* = .12, *t* = -5.439, *p* < .000; for coping, *a*_3_ = -.63, *SE* = .15, *t* = .097, *p* = .923; for time spent studying, *a*_3_ = -375.28, *SE* = 291.60, *t* = -2.593, *p* = .010). Curvature along the line of incongruence for all three outcomes was not significant (for focus, *a*_4_ = .32, *SE* = .36, *t* = .874, *p* = .383; for coping, *a*_4_ = .03, *SE* = .30, *t* = .097, *p* = .923; for time spent studying, *a*_4_ = 143.95, *SE* = 291.60, *t* = .494, *p* = .622), indicating that the direction–but not the degree–of the discrepancy between anticipated and experience PA translates into meaningful increases in these outcomes. In sum, these results support both the congruence and positive incongruence propositions for PA.

The response surfaces for NA predicting time spent studying is shown in Fig 7. Per Shanock et al. [30], we did not create response surfaces for NA predicting coping and focus because the *R*^2^ value for these regression analyses was not significantly different from zero. For this outcome, the line of agreement indicates that, in support of the congruence proposition, time spent studying is higher when both anticipated and experienced NA are high versus when both predictors are low (*a*_1_ = 273.74, *SE* = 89.27, *t* = 3.066, *p* = .002). Thus, people spend more time studying when they anticipate feeling—and ultimately feel—more negatively while studying. We return to this finding in the Discussion section. The curvature of this line is not significant, meaning that the relationship is linear (*a*_2_ = 94.94, *SE* = 65.12, *t* = 1.458, *p* = .147). Further, the line of incongruence for NA and time spent studying (*a*_3_ = -224.17, *SE* = 191.14, *t* = -1.173, *p* = .242) and its curvature (*a*_4_ = 7.91, *SE* = 343.67, *t* = .023, *p* = .982) were not significant. These nonsignificant findings for *a*_3_ and *a*_4_ mean that, in study 2, we failed to find support for the incongruence proposition for NA predicting time spent studying.

**Fig 7:** Response surface area wherein time spent studying is predicted by anticipated—experienced negative affect discrepancy (Study 2).

### Study 2 discussion

Study 2 extended study 1 by evaluating how affective forecasts relate to more proximal indicators of performance (i.e., goal-directed behaviors). As in study 1, affective forecasts were fairly accurate, both in terms of magnitude and direction. Also consistent with study 1, affective experiences that are anticipated to be, and experienced as, more positive tend to be associated with higher levels of goal-directed behaviors. Furthermore, these outcomes are enhanced when people experience greater levels of PA than anticipated. Taken together, Study 2 provided additional support for the congruence and positive incongruence propositions for PA. With regard to NA, in Study 2 we again found support for the congruence proposition; however, in Study 2 we found that time spent studying was enhanced when NA was anticipated to be *high* and then was experienced as high. Moreover, we failed to find support for either incongruence proposition for NA because goal-directed behaviors are not significantly enhanced further when there is a discrepancy between anticipated and experienced NA.

## General discussion

The purpose of the current work was to investigate affective forecasting in self-reported task performance. Scholarly interest regarding the importance of emotion in learning and performance contexts has grown dramatically over the past two decades [37]. Despite this flurry of research, there remain many unchartered paths about the occurrence and potential impact of affective phenomena in task performance. We see future-oriented affective thinking as one such area ripe for study in this domain.

Additionally, by exploring affective forecasting in the context of (self-reported) task performance, a second intended contribution of these studies was to contribute knowledge to the affective forecasting literature. As noted in the beginning of the paper, the current investigation was different from the typical study in this research area in various respects. This divergence provided the opportunity to address the generalizability (or boundary conditions) of foundational results and suggest future directions stemming from discrepancies in results. Below, we review the key study findings, discussing similarities and differences with past affective forecasting research, and offering future scholarly directions.

### Effects of affective forecasts on self-reported performance and goal-directed behaviors

The major research topic addressed here was how affective forecasts mesh with in-the-moment affect to influence self-reported task performance. Broadly speaking, these findings are consistent with the notion that prospective thinking is prevalent because of its functionality (e.g., [27]). Such thinking can involve simulating future events and their contingencies [14]. Affect seems to be a key ingredient in this process by providing the potential incentive or deterrents of potential actions and, as such, guiding decision-making making about alternative courses of action.

First, with regard to the significance of *anticipated affect* specifically, our results are consistent with a meta-analysis showing that anticipated affect predicts behavior especially well—in fact, perhaps better than in-the-moment affect [15]. The current results demonstrating the role of anticipated affect imply scholars need to pursue a different (additional) avenue in the study of affect and performance. In the organizational context, relevant accounts almost exclusively have addressed in-the-moment affect impacting performance (e.g., [38]). Often, these explanations prioritize affect emanating from the task characteristics (e.g., difficulty, workload) as impacting proximal cognitive and motivational antecedents of performance (e.g., [25]). With a few notable theoretical exceptions, though (e.g., [25, 39]), the potential importance of anticipated affect has received almost no attention in the organizational arena.

The second conclusion that seems particularly notable concerns the nature of the effects. In general, anticipating the performance episode to be more affectively pleasant (i.e., characterized by higher PA and lower NA) was associated with better self-reported task performance. To help move theory forward, we consider this finding in relation to research on positive emotions about the *outcomes* of actions. Research has shown that *fantasizing* about positive outcomes is not sufficient to bring about those desired ends and, in some cases, may even undermine the behaviors necessary to achieve them [40]. In order for those fantasies to translate into valued outcomes (e.g., health and interpersonal outcomes in their studies), one also must engage in mental simulation about the process of achieving those outcomes (e.g., addressing potential obstacles; see [41]).

The current study was about the affect associated with that mental simulation of *process*. But our findings seem consistent with those on fantasizing—and appear to fill part of the theoretical picture about how forecasting impacts performance (as measured here by self-reports). In particular, the findings that feeling better than anticipated was associated with the highest levels of self-rated performance may imply that the most effective simulations incorporated potential challenges (not all of which were realized). Thus, just as fantasizing without consideration of the process will not yield the largest performance gains, neither will too favorable of affective forecasts about the process.

This notion would seem to have important practical implications. The intuitive advice to “be positive” about upcoming tasks, or the notion that leaders should use motivational language emphasizing how good employees will feel upon achieving success may be misguided. Positive affect can enhance various motivational perceptions such as self-efficacy [42] and task-related valence, instrumentality, and expectancy [43]. However, unless those perceptions are paired with realistic simulations about the process of task engagement, performance ultimately may not improve. Our findings, paired with the past ones noted above, suggest utility in fostering simulations about task engagement. Affective expectations about task engagement should be only as positive as the simulations realistically allow, and perhaps less favorable than they allow.

### The (in)accuracy of performance-related affective forecasts

Although not the primary focus of this research, the two studies presented here are among the only investigations we are aware examining the accuracy of performance-related affective forecasts. Perhaps more significantly, the current findings bear mention because they partly differ from those found in studies of affective forecasting about discrete decisions or outcomes (e.g. [44, 9]).

In contrast to those past results, our results did not show a systematic tendency to foresee task performance episodes as either more positive or more aversive than they later turned out to be. We see two explanations for this seemingly divergent conclusion as especially plausible. One possibility is that, unlike rare events about which participants are often asked to make forecasts (e.g., being assigned to a more or less desirable housing dormitory [9]), participants here made forecasts about familiar activities. According to this explanation, the normal distribution of inaccuracies reflects errors in foreseeing specific (sometimes unknowable) contextual details (e.g., who would be present) rather than to a psychological tendency to under- or over- estimate one’s capacity to adjust to the occurrence (see [45]).

However, further findings suggest that the greater familiarity of these occurrences was not responsible for these findings. Specifically, results from an additional exploratory analysis (using General Estimation Equations to account for the nesting) with the Study 1 data showed that familiarity (with the chosen task activity) did not significantly predict accuracy (i.e., absolute discrepancies) for positive affect (level (*b* = -.003, *SE* = .02, χ^2^ = .02, *p* = .899) or negative affect (*b* = -.001, *SE* = .02, χ^2^ = .004, *p* = .952). That is, greater familiarity was not associated with more accurate forecasts. Of note, participants were told that they could choose activities that are “typical, regularly occurring as part of your work” or events that “might be more unusual and/or infrequently occurring.” Descriptive statistics confirmed that there was indeed a range of familiarity for the reported activities. Thus, these null results do not appear to be due to restricted variance of familiarity.

The other possibility that seems most plausible to us is that these task activities are associated with a different type of both anticipated (and experienced) affect than are discrete decisions and strong affective events. For most task activities, affect appears to take the form of a more mild or ambient state or “sense” of how one feels [46]. In contrast, important decisions or salient events tend to produce strong discrete emotional reactions [47]. Borrowing from the language of affective events theory, workdays may be thought of as a series of performance episodes (e.g., meeting with a supervisor followed by a two-hour shift, etc. [48]). Affective events may punctuate these episodes, but they would seem less likely candidates for affective forecasts due to their mainly being unexpected (see [39]). Future research explicitly testing which aspects of performance episodes distinguish affective forecasting in regard to them, versus about discrete affective events—thus would seem valuable.

### Boundary conditions and limitations

Several aspects of the study designs vis-a-vis the results warrant mention. At a general level, we note that designing a study on affective forecasting necessitates making a series of methodological choices, the decisions about which ultimately may influence the study findings. While we asked about affect in specific task scenarios at a given time on a given day, another option would have been to elicit predictions about work or studying (“in general”). Plausibly, this latter approach may have drawn more on semantic, rather than episodic, retrieval and, correspondingly yielded different affective forecasts [49]. To the extent that there does exist amongst people a pervasive negative schema of work, its influence perhaps would have been more evident using that approach (see [50]). In turn, affective forecasting may have been far less accurate. Also, related to a point above, we perhaps could have demonstrated lower accuracy if we had asked participants to consider particularly affectively-laden events, such as upcoming meetings with leaders or interactions with hostile customers [51]. To the degree that seemingly dramatic events are not as emotional as anticipated, accuracy again would suffer.

Instead of adopting these approaches, we took a rather conservative strategy. If performance-related affective forecasting is accurate much of the time, it should (and largely did) manifest with the current design. Studies using different verbiage and designs to examine the generalizability of the current findings, though, are certainly important next steps. In particular, we would advocate for qualitative or mixed-methods studies that aim to capture the occurrence and nature of real-time affective prospection about work. Thought-sampling studies would seem well-suited to capture these naturalistic thoughts, and methodologies such as cognitive interviews would be useful in probing them.

Another subject that warrants discussion is the specificity of the affective forecasts we collected in these studies. As a Reviewer noted, the current design does not wholly allow for disentangling affect about engaging in the task from affect felt when the task is completed. When asking people to report their anticipated affect about engaging in such tasks, we certainly are capturing affective forecasts about how people will feel while progressing toward task completion. We also may be capturing anticipated feelings upon having completed the task, given the nature of the tasks under investigation. In both studies, we collected data about prolonged behaviors that do not have outcomes. As an example, two Study 1 participants reported cleaning bathrooms and reviewing documents, respectively. For such effortful, prolonged tasks, their execution is one-in-the-same as their (likely primary) outcome–progressing toward completion. For these types of tasks, we likely were tapping into anticipated affect, both in terms of how people would feel while engaging in the task as well as the affect people anticipated feeling when they complete the task. This scenario becomes even more complex when execution of the task would coincide with other outcomes that may have emotional valence (e.g., promotions, positive or negative feedback etc.). While the tasks reported in Study 1 (and studying in Study 2) do not have obvious links to immediate, highly valued outcomes, there certainly remains the possibility that cognitions about those externalities also influenced anticipated affect during task execution. This said, whether or not distilling the unique contributions of these sources of affective forecasts is methodologically feasible–or conceptually desirable–remains an open question in our view.

In a similar vein, the inability of the current study designs to capture the temporal ordering of experienced affect vis-a-vis perceived performance also warrants mention. Although we positioned affect as an antecedent to performance, reality often may be more dynamic and complex than this ordering suggests. Most likely, anticipated affect partly reflects predicted performance. Similarly, reports of experienced affect partially may reflect perceived performance on the task in which one is engaged (or did just engage). These notions may explain the Study 2 findings in which time spent studying was positively related to both anticipated and experienced negative affect. People may have predicted feeling worse because they recognized they would have to study longer and then did indeed feel worse after doing so.

Indeed, the real-time relationship between experienced affect and perceived success may follow various dynamic trajectories. For instance, positive affect may beget perceived success which may beget more positive affect, etc. (e.g., [52]). Seen in this way, attempts at disentangling the causal ordering may not, in fact, be very realistic. Both from a phenomenological perspective and a practical one, attempting to separate components that are linked during real-time performance may prove a largely futile endeavor. This said, insofar as achieving this separation is realistic, we would suggest that controlled experiments would be the preferred method to achieve this end. Specifically, controlling (or manipulating) either felt affect or, perhaps more realistically and useful, the amount or valence of task feedback—seems like a promising paradigm to use in investigating this issue.

Lastly, we relied on relatively subjective measures of task performance due to the nature of the tasks being studied (i.e., those that require prolonged effort and without clear outcomes). Hence, we used the term self-reported performance. For these types of tasks (e.g., reviewing reports in study 1, and studying for an exam in study 2), meaningful objective measures appeared elusive. Therefore, consistent with best practices for assessing performance, we relied on behaviorally-based subjective measures in study 2 (e.g., time spent studying, learning-oriented coping behaviors). (Exam scores were not evaluated as an objective measure in study 2 because again, we were interested in understanding how students’ affective discrepancies influenced how they would perform while studying for the exam–not while taking the exam.) In study 1, participants held multiple types of jobs and therefore were reporting a wide variety of different types of work tasks/activities. Therefore, we used a more general subjective measure of performance widely applicable to all of the work tasks reported by study 1 participants. Future studies should consider incorporating relatively objective measures to capture the full spectrum of the performance domain as appropriate.

## Conclusion

The findings from these two studies suggest significant utility in continuing to examine affective forecasting in the task performance domain. Results showed that anticipating greater positive affect and lower negative affect generally was associated with higher self-reported performance. Furthermore, feeling better than predicted during the task was associated with additional gains in self-reported performance. Findings also showed that forecasts about task episodes varied in accuracy but did not conform to the distribution found in other affective forecasting research (about discrete events or decisions). Our hope is that this foundational work will engender subsequent efforts to explore the nature and implications of affective forecasting in the organizational arena.
